The article "Influencing Factors of College Students' Use of Sports Apps in Mandatory Situations: Based on UTAUT and SDT" was published in 2022. Journal: Biomed Res Int.

# Influencing Factors of College Students' Use of Sports Apps in Mandatory Situations: Based on UTAUT and SDT

**DOI:** 10.1155/2022/9378860

**Published:** 2022-09-22

**Authors:** Jian Guo

**Affiliations:** Department of Physical Education, Liaoning University of Technology, Jinzhou 121001, China

## Abstract

Sports apps are third-party applications for smartphones or wearables that can help users record fitness data and guide their exercise behavior. Many Chinese college students are compelled to use sports apps for running exercises to improve their physical health and cultivate extracurricular exercise habits; however, the acceptance and use of sports apps by college students in mandatory situations requires elucidation. We explored the influencing factors of university students' behavioral intention and usage behavior to use sports apps in mandatory situations by combining the unified theory of acceptance and use of technology and the Self-Determination Theory. A questionnaire survey was conducted among 249 students of Liaoning University of Technology by using non-probabilistic convenient sampling. Data analysis was performed by employing partial least squares structural equation modeling. The results showed that (1) the research model explained 66% (*R*^2^ = 0.66) of the variance in behavioral intention and 30% (*R*^2^ = 0.30) of the variance in usage behavior; (2) performance expectancy, effort expectancy, social influence, and autonomous motivation significantly positively affected behavioral intention, while controlled motivation negatively affected behavioral intention; and (3) behavioral intention, autonomous motivation, and controlled motivation significantly positively affected usage behavior. The influence of facilitating conditions on usage behavior was non-significant. The results will help technical developers and schools to better understand the influencing factors of college students' use of sports apps in mandatory situations, and formulate corresponding improvement strategies and policies to further promote the role sports apps play in college students' exercise behavior.

## 1. Introduction

Smart phones and mobile Internet have been popularized in China with the development of science and technology. The latest survey report [1] shows that the total number of mobile Internet users in China reached 1.029 billion by the end of 2021, and mobile Internet access traffic had reached 221.6 billion GB in 2021, an increase of 33.9% over the previous year. Concurrently, the use of apps is escalating, as well. By 2021, the total number of on-shelf apps distributions in third-party app stores reached 2.1072 trillion, an increase of 31% compared with the same period the previous year. In this context, sports apps—born from the combination of sports, smart phones, and mobile Internet—have a broader space for development.

Sports apps are third-party applications for smartphones or wearables that can help users record fitness data, guide learning in sports, and lead healthy lifestyles [2]. With the rapid development of sports apps, there have been some challenges [2–4], such as serious content homogenization; lack of service model innovation; lack of data analysis ability; difficulty formulating a scientific and targeted training guidance program; and a functional design that targets young people but fails to address the unmet exercise needs of the middle-aged, elderly, and special groups. Nevertheless, sports apps have been widely used to improve exercise behavior and health management, greatly contributed to the reduction of global obesity rate and medical costs [5], because they incorporate individualized physical activity behavior modification technologies such as self-monitoring, goal planning, and performance feedback [6]. Research shows that in addition to significantly improving and maintaining users' level of physical activity [7, 8], sports apps enable users to overcome exercise obstacles, participate in higher-intensity physical activities [9], and improve their exercise attitude and behavior habits compared with non-users [10]. College students form a key group of users of smart phones and sports apps [6, 11, 12] as they satisfy their exercise demands and improve their health status [12, 13].

An increasing number of college students are sedentary and lack physical activity, and their physical health is worrying [14]. This may be owing to addiction to mobile devices and online games during periods for extracurricular activities [15]. Numerous schools and universities in China compel students to run on campus using sports apps such as “Sports World Campus,” “Trail Running,” and “Seeking Campus” to enhance their physical health and develop extracurricular exercise habits [16]. This kind of behavior plays a positive role in improving students' physical health during the school period [17, 18]. However, many students do not agree with the school's behavior of compelling them to use sports apps for physical exercise [16, 19], because the school prescribes the route, mileage, and running times when students use the apps, and the running completion has a great impact on the final results of physical education. Some studies [20] have shown that users will not use it actively and efficiently if they are compelled to accept and often use a certain technology or system. Similarly, if students are compelled to run, although they will accomplish the school's objectives, they may do so with negative feelings such as resistance and grumbling, which will ultimately go against the school's original mission. This is detrimental to the development of students' exercise routines and long-term health awareness. Sports apps can play a completely positive role when they are widely accepted and used by students. Therefore, it is necessary to study the influencing factors of college students' intention and behavior to use sports apps in mandatory situations.

Furthermore, taking the influencing factors of compelling college students to accept and use sports apps as the theme of this study is also based on the following two reasons. On the one hand, the mandatory behavior of the school has played a positive role in promoting the exercise behavior of college students. The research shows that using modern information technology to compel students to run can not only effectively increase the time and frequency of students' extracurricular exercise [18], but also strongly promote and effectively supervise the improvement of college students' physical health and the cultivation of exercise habits [15]. On the other hand, in mandatory situations, there are some differences in students' motivation to use sports apps [21], and there are still some deficiencies in the management and maintenance of sports apps and so on [22]. The conduct of this study can identify the positive and negative factors that affect college students' acceptance and use of sports apps in mandatory situations, provide reference for technical developers and schools, and further promote the application of sports apps in college students' exercise behavior.

Focusing on the theme of college students' use of sports apps, researchers have conducted relevant research using quantitative [11, 12], qualitative [13, 23], and mixed research methods [24]. However, these studies were based on voluntary situations for personal sports and health purposes. At present, only a few Chinese scholars have studied the influencing factors of college students' use of sports apps in mandatory situations. For example, Xu [25] and Wang et al. [16] used qualitative methods to conduct research from the viewpoint of media characteristics and health communication psychology. Presently, quantitative research based on theoretical models is sparse.

This study will conduct quantitative research based on theoretical models. The unified theory of acceptance and use of technology (UTAUT) is a model widely used in technology acceptance research [26]. This study chooses UTAUT as the theoretical basis for three reasons. First, many early studies, especially those based on the technology acceptance model (TAM) and its derivative models, were performed in user voluntary situations, while researchers commonly questioned the efficacy of applying the traditional technology acceptance model in mandatory situations [20, 27, 28]. Venkatesh et al. [26] considered the usage situations (voluntary and mandatory) when creating the UTAUT. Therefore, UTAUT is applicable to the mandatory situations of this study. Second, the UTAUT was developed to integrate information and communication technology (ICT) research and theory into a comprehensive theoretical model [26, 29], while sports apps are products of ICT. Furthermore, other studies [11, 30, 31] have demonstrated the value of the UTAUT and its expanded model in the research of sports apps. Third, the UTAUT integrated the core elements of eight models and theories when it was created. While keeping a simple structure, the model explains as much as 70% of the variance in intention and 50% of the variance in behavior to use technology, which is a considerable improvement above any of the previous eight models and their expansions. A meta-analysis also indicated that UTAUT is an effective and robust model based on ample empirical evidence [32]. The above reasons and arguments convince us that UTAUT is an appropriate theoretical model and can lay a theoretical foundation for this study.

User acceptance and usage of technology is a complicated mechanism, and a single theory or model's explanatory capacity is limited; hence, it is necessary to incorporate extra external variables or combine UTAUT with other theories to boost the model's explanatory power [33, 34]. Furthermore, the UTAUT model, according to Dwivedi et al. [35], excludes a crucial component: the personal characteristics that influence behavior, particularly the neglect of individual psychological variances including basic psychological requirements and motivation [33]. Moreover, the individual difference of motivation is an important determinant of technology acceptance success [36]. Several researchers in information systems urge the need to include motivational factors to explain the acceptance and use of information technology [37, 38]. Self-Determination Theory (SDT) is a macroscopic theory used to explain human behavior and motivation [39]. Therefore, the combination of SDT and UTAUT as the theoretical framework of this study can make up for the limitations of UTAUT and improve the accuracy and comprehensiveness of the research findings.

SDT is used in this study for three reasons. First, SDT has been applied in the design of sports apps owing to the rapid growth of communication technology and mobile Internet. Research shows that sports apps designed and developed according to SDT can better meet users' basic psychological needs and improve their intrinsic motivation for exercise [29]. Second, researchers have applied SDT to the related research on sports apps and achieved notable results. For example, Choi et al. showed that whether sports apps can meet the basic psychological needs of users for exercise is crucial for users to perceive the usefulness and utilization of sports apps [40]; Molina et al. found that users' motivation to use apps will shift from extrinsic motivation to intrinsic motivation with the exercise effect brought by sports apps to users [41]. Third, other studies have tried to combine SDT with the TAM and the expectation confirmation model to study the acceptance and use of sports apps and mobile health apps, and they indicated the effectiveness of SDT in technology acceptance related models [42, 43]. At present, few researchers have combined UTAUT and SDT to study the acceptance and use of sports apps; thus, a research gap exists in mandatory situations.

The “Sports World Campus” app (hereafter referred to as “campus running” app) is a widely used sports app on university campuses in China, and numerous universities compel students to use this app for running exercise [16]. Therefore, the wide compulsory use of “campus running” app provides a good practical basis for filling the gap in the research on the influencing factors of using sports apps in mandatory situations. This study constructs a research model based on UTAUT and SDT, taking the “campus running” app as an example, and it reveals the factors influencing college students' acceptance and use of sports apps in mandatory situations, to fully reflect the positive role of new media technology in affecting college students' physical activity habits and improving their physical health.

First, according to UTAUT (Figure 1), performance expectancy, effort expectancy, and social influence directly affect behavioral intention. Facilitating conditions and behavioral intention directly affect use behavior. Gender, age, experience, and voluntariness of use are the four moderating variables of the model. Based on UTAUT [26] and related research of sports apps [11, 30, 31], we hypothesized that performance expectancy (H1), effort expectancy (H2), and social influence (H3) will have significant positive effects on students' behavioral intention to use the “campus running” app. Facilitating conditions (H4) and behavioral intention (H5) will have significant positive effects on students' use behavior of the app. Owing to the fact that the “campus running” app is mandatory and the participants were freshmen and sophomores, the differences in their age and operational experience will have no effect on the results [11]. Consequently, this study retains gender alone as the moderating variable. Therefore, we hypothesized that the influence of performance expectancy (H6a), effort expectancy (H6b), and social influence (H6c) on behavioral intention will be moderated by gender.

Second, SDT classifies motivation into autonomous motivation and controlled motivation according to the degree of autonomy or control [39]. Autonomous motivation is an important driving factor of behavior since it can meet the needs of individual autonomy. Therefore, we hypothesized that autonomous motivation would have significant positive effects on both intention (H7a) and behavior (H7b) to use the “campus running” app. Controlled motivation has less effect on exercise intention and behavior [44], and it has a dual effect of stimulating students' liveliness and placing them under psychological pressure [45]. Therefore, we hypothesized that controlled motivation would have no significant effects on both intention (H8a) and behavior (H8b) to use the “campus running” app. The final research model is shown in Figure 2.

Finally, this study used the “campus running” app as an example. This app is a sports software developed by China Zhejiang Wanhang Information Technology Co., Ltd. for college students. In addition to specifying students' running route through the fixed-point clock-in function, it also sets students' running speed and mileage. It can upload the running data to the “cloud” monitoring platform after students have finished running and can help physical education teachers to supervise and monitor students' exercise behavior. It has the following advantages compared with similar apps such as “Trail Running” and “Seeking Campus.” The first is its rich functions. In addition to the functions of exercise and supervision, the app also has a perfect “community” function for students to publish “sports mood” and has interactive functions such as like and comments. Second, it has the largest number of student users. Since this app is free for all colleges and universities to use and operates stably, it has been extended to nearly 500 university campuses in 26 provinces and cities in China by 2020 [16]. It has the most student users compared with similar app in China. Third, its validity has been tested. The research of Meng et al. [18] and Yang et al. [17] shows that this app plays a positive role in enhancing students' physical health and cultivating students' exercise habits during school. Therefore, the college students who use the “campus running” app as the survey object have a certain representativeness and universality.

## 2. Materials and Methods

### 2.1. Ethical Statement

This study was approved by the Ethics Committee of Liaoning University of Technology (no. 20210503). All participants were given a brief introduction to the study and informed of its purpose, as well as declarations of anonymity and confidentiality before participating, and they provided informed consent. We conducted this study in accordance with the latest revised ethical guidelines of the Declaration of Helsinki.

### 2.2. Power Calculation

Before recruitment, a power calculation was conducted to determine the required sample size. According to the suggestion of Hair [46], the sample size was calculated following Cohen's recommendations for multiple ordinary least squares regression analysis [47]; one would need 84 observations to achieve a significance level of 5% and a statistical power of 80% for detecting *R*^2^ values of at least 0.25 (with a 5% probability of error). A total of 249 participants were recruited, which was greater than the minimum value of 84, meeting the study requirements.

### 2.3. Measurement Instrument

To evaluate the theoretical model's hypotheses, a survey was conducted that included items for all the model's constructs, as well as grade, gender, age, physical condition, and the last six digits of the student ID (used to match the usage behavior of the “campus running” app). The survey consisted of 25 items and assessed seven study constructs: performance expectancy, effort expectancy, social influence, facilitating conditions, autonomous motivation, controlled motivation and behavioral intention. The scale items, such as performance expectancy, effort expectancy, social influence, and facilitating conditions, were adapted from the questionnaires developed by Venkatesh [26], Liu [11], and Yang [30]. The motivation scale items were adapted from the behavioral regulation in exercise questionnaire (BREQ-3) developed by Markland et al. and Wilson et al. [48, 49]. The scale BREQ-3 is available free of charge on the website of the Exercise Motivation (authorized by the author). All items were measured on a seven-point Likert-type scale ranging from 1 = strongly disagree to 7 = strongly agree. The intention to use the “campus running” app was measured by three fill-in-the-blank questions: “how many times do you intend/plan/try to use ‘campus running' app in the next week?” The usage behavior of “campus running” app was measured by the number of actual uses within seven days after completing the questionnaire. These usage behavior data were exported directly from the app's data monitoring platform. Furthermore, to mitigate the impact of language differences, the English scale has been translated and culturally adjusted strictly following the Beaton cross-cultural adaptation guidelines [50], and adopting the steps of literal translation, back translation, integration, expert consultation, pre-investigation, and formation of preliminary tools.

### 2.4. Participants

Participants included freshmen and sophomores at the Liaoning University of Technology. This university is one of the first schools to compel students to use sports apps for running exercise and has compelled students to use the “campus running” app for four consecutive years. The school's sports department has a relatively perfect system related to “campus running.” Students' experience and cognition of the “campus running” app are extensive and constant, and responses to the questionnaire are typical. The university compels all freshmen and sophomores to use the “campus running” app every semester. Therefore, the data from the survey of freshmen and sophomores who are using the “campus running” app are authentic. At present, there is no such thing as giving up studies or other unfavorable things because the school compels students to use the app.

The inclusion criteria for participants were being freshmen or sophomores, healthy and without disability, able to use the “campus running” app as required by the school, volunteering to participate in this study, and signing an informed consent form. A total of 350 questionnaires were distributed and 343 questionnaires were collected. In the screening of questionnaires, 94 unqualified questionnaires were excluded according to the following criteria: (i) the last six digits of the student ID were filled incorrectly; hence, the relevant usage behavior data cannot be found on the app's data monitoring platform; and (ii) students missed the key items in the questionnaire. Finally, 249 valid questionnaires were obtained, and the effective recovery rate was 72.59%. The mean age of participants was 19.28 (SD = ±1.02) years. Most were female (58.23%) and freshmen (53.01%). In addition, 48.19% of the participants used the “campus running” app 4–5 times a week (Table 1).

### 2.5. Procedure

We employed non-probabilistic convenient sampling to distribute paper questionnaires (Table 2) at different locations on campus (such as the entrance of classrooms and canteens). All questionnaires were distributed and collected on the spot on May 10, 2021. All questionnaires were collected on the spot. Before the questionnaires were distributed, the investigators introduced the purpose of the survey to each participant and assured them that their information was confidential. In order to ensure the veracity and completeness of the questionnaire information, the researchers examined the contents of the questionnaires one by one after collecting them, and excluded the questionnaires with obvious logical errors and missing the key items. The two people checked together when entering the questionnaire data, and used SPSS 20.0 to check whether there are extreme values, normal distribution and so on.

### 2.6. Statistical Analysis

We used SPSS 20.0 to perform descriptive statistics on participant and data characteristics, and we used SmartPLS3.3.3 to evaluate the measurement model and verify the structural model. The research model is a more complex and exploratory model with moderating variables. Therefore, the research model was tested using the partial least squares structural equation modeling (PLS-SEM) approach. PLS-SEM, in addition to being used to test the model's complex causality [51], has a greater statistical power at all sample sizes, and there are no strict requirements for the distribution of data [52]. As shown in Table 2, the data of this study are normally distributed.

According to the suggestion of Hair et al. [46], the study analyzed the survey data in two steps. The first stage involved validating the measurement model, and the second stage examined the latent variables' structural relationships. We first established the measures' reliability and validity before evaluating the research model's structural relationship.

## 3. Results

### 3.1. Measurement Model

After preliminary test, it was found that the factor loadings (FL) of all items were greater than 0.70, except for CM4 (0.67) and AM6 (0.54) (Table 2). Therefore, items CM4 and AM6 were removed according to the suggestion by Hair et al. All items of autonomous motivation and controlled motivation were packaged into 3 items and 2 items, respectively, using the theoretical packing method.

To evaluate the measurement model of reflective constructs, this study examined their internal reliability, convergent validity, and discriminant validity. As shown in Table 3, the composite reliability and the Cronbach's alpha of all constructs were greater than 0.70, as suggested by Hair et al. [46]. Therefore, the measurement model showed strong internal consistency reliability. To determine convergent validity, the average variance extracted (AVE) and FL were used; all estimated FL and AVE values for each construct should be greater than 0.70 and 0.50 [46]. The results indicated that the FL of each item in the measurement model, which ranged from 0.78 to 0.93 (Table 4), fulfilled the rule of thumb of Hair et al. [46]. The AVEs of all constructs in this study ranged between 0.64 and 0.81 (Table 3), which is greater than 0.50, indicating a construct's ability to explain 50% of the variation of its indicators; hence, the measures exhibit good convergent validity. In addition, two measures of discriminant validity have been proposed [46]. One method is to examine the cross loadings of the indicators. Specifically, an indicator's outer loading on the associated construct should be greater than all of its loadings on other constructs. As illustrated in Table 4, these indicators have a higher loading on their own construct than on others. The Fornell-Larcker criterion is a second and more conservative approach to assessing discriminant validity. According to the criterion, a latent construct has a higher correlation with its own indicators than it does with any other indicator in the model. As shown in Table 3, the values on-diagonal values are greater than off-diagonal values. Therefore, the model has good discriminant validity.

### 3.2. Structural Model

After determining the validity of the measurement model, we used the structural model to test the hypotheses. The research model's explained variance (*R*^2^) values for the behavioral intention and usage behavior of “campus running” app were 0.66 and 0.30, respectively. This shows that the research model can explain 66% of the variance in behavioral intention and 30% of the variance in usage behavior associated with the “campus running” app. Along with *R*^2^ values, effect size (*f*^2^) is used to determine whether an independent variable has a significant effect on a dependent variable. According to Cohen's (1988) standard, the results indicate that the *f*^2^ values for the supported hypotheses are acceptable (Table 5). The predicted relevance (*Q*^2^) value is also evaluated by running the blindfolding procedure and calculated using the cross-validated redundancy approach. According to Chin [53], a *Q*^2^ value greater than zero indicates that the model is predictively significant. The results show that *Q*^2^ values of behavioral intention and usage behavior are 0.44 and 0.28, respectively. This indicates that the structural model is sufficiently predictive.

The significance levels of the path coefficients were checked using the nonparametric bootstrapping procedure with 5000 iterations [46]. The results indicated that performance expectancy (*β* =0.33; *p <0.001*), effort expectancy (*β* =0.33; *p <0.001*), social influence (*β* =0.22; *p <0.001*), and autonomous motivation (*β* =0.19; *p =0.008*) all positively affected behavioral intention, while controlled motivation (*β* = -0.10; *p =0.050*) negatively affected behavioral intention. Behavioral intention (*β* =0.21; *p =0.006*), autonomous motivation (*β* =0.27; *p =0.006*), and controlled motivation (*β* =0.16; *p =0.034*) positively affected usage behavior, while the influence of facilitating conditions (*β* = -0.03; *p =0.694*) on usage behavior was non-significant. Consequently, H1–H3, H5, H7a, and H7b were supported, while H4, H8a, and H8b were rejected (Table 5, Figure 3).

Following validation of the main model, the moderating effect of gender was examined using the multi-group analysis function of the SmartPLS software. The results indicate that the influence of performance expectancy, effort expectancy, and social influence on behavioral intention were not regulated by gender. Consequently, H6a-H6c were rejected.

## 4. Discussion

The purpose of this study is to examine the influencing factors of university students' behavioral intention and usage behavior to use sports apps in mandatory situations from the perspectives of technology acceptance and motivation. The participants were all from Liaoning University of Technology in China, which is one of the first schools to compel students to use sports apps for running exercise, and the sample size through power calculation met the needs of the study. Therefore, the research findings have certain generalizability and representativeness. The findings indicated that the research model in this study can explain 66% of the variance in behavioral intention and 30% of the variance in usage behavior to use sports apps in mandatory situations. Performance expectancy, effort expectancy, social influence, and autonomous motivation are positive factors of behavioral intention, while controlled motivation is a negative factor. Behavioral intention, autonomous motivation, and controlled motivation are positive factors of usage behavior, while the influence of facilitating conditions on usage behavior is non-significant (Figure 3). The main findings are discussed as follows.

### 4.1. Principal Findings

In this study, both performance expectancy and effort expectancy significantly positively affected participants' behavioral intention to use sports apps, and the effects were similar. This finding is slightly different from previous research findings. Chang et al. [54] believed that new technologies and systems will be the only way for users to complete daily tasks, and employees will pay more attention to the usefulness of the system in mandatory situations. Consequently, performance expectancy has a greater impact on behavioral intention than effort expectancy does. However, students exercise not only through sports apps, but also through other extracurricular activities that can help them improve their physical quality. This may weaken the effect of performance expectancy on behavioral intention. Additionally, the sports apps use GPS [25] and students are compelled to clock-in at a fixed point. The campus network signal, building environment, weather conditions, mobile phone performance, and brands affect the timeliness of clocking-in for sports apps, and the school has a strict time limit for students to complete the running task. Consequently, students may have been more concerned with the smoothness of the clock-in process than with the exercise function of the sports apps. Therefore, the technical developers of sports apps such as “campus running” need to maintain the basic exercise function of apps and focus on improving the acceptability of apps' GPS signal and its compatibility with different brands of mobile phones to ensure the timeliness of students' successful clocking-in, to enhance students' intention to use sports apps.

Social influence significantly positively affected behavioral intention. Although this result is consistent with the findings of Liu et al. [11] and Ndayizigamiye et al. [31] in voluntary situations, the influence mechanism of social influence on behavioral intention differs across distinct situations (voluntary and mandatory). Hwang et al. [27] argued that social influence affects behavioral intention through three mechanisms: compliance, internalization, and identification. Social influence in voluntary situations affects people's perception of technology through internalization and identification, while in mandatory situations, compliance is the main influence mechanism of social influence on behavioral intention. Individuals are more likely to comply with the expected behavior of others when the person or organization who implements the compelled behavior has the ability to reward or punish the expected behavior [26]. The school compels students to use the sports apps for physical exercise, and the relevant sports departments or physical education teachers have the ability to reward or punish (add or deduct points for final physical education scores) the students according to their running completion. Consequently, students are more likely to follow the recommendations and requirements of their teachers to exercise using the sports apps. However, the impact of social influence on behavioral intention may also diminish when the rewards or punishments disappear. Therefore, it is necessary to develop appropriate strategies to promote the gradual internalization of compliance into internalization and identification. For example, we can strengthen the construction of the community within the sports apps to promote the social interaction of sports among students or set-up a daily running mileage ranking in the community to influence the surrounding students by the power of example.

In the mandatory situation, autonomous motivation significantly positively affected behavioral intention and usage behavior of using sports apps. Furthermore, the effect of autonomous motivation on usage behavior was higher than behavioral intention. According to SDT [39], the behaviors engaged in by individuals with autonomous motivation are self-determined (autonomous), which are more aligned with the needs of individual autonomy, and have a positive impact on both intention and behavior. Hagger et al. [44] showed that autonomous motivation has a significant positive effect on the intention and behavior of a variety of health-related behaviors and is not affected by individual differences. Behavioral intention has been shown to be the strongest determinant of the usage behavior of technology [55, 56]. However, the results indicate that the effect of behavioral intention on usage behavior is less than autonomous motivation in the mandatory situation. The reason may be that the influence of intention on behavior can be influenced by the behavioral situations (voluntary or mandatory). In voluntary situations, the user can use their free will to fully control their behavior; that is, they have will control which can moderate the relationship between intention and behavior. The stronger the will control, the greater influence of intention on behavior [57]. However, in mandatory situations, the user perceives lower will control, which will weaken the influence of intention on behavior. Contrastingly, the positive effects of autonomous motivation on behavior may not be influenced by the behavioral situations. In this study, students with autonomous motivation realized the health value brought by the mandatory behavior of the school or meet their intrinsic need for exercise. Consequently, students with autonomous motivation will respond more positively to the school's mandatory behavior and are more likely to adhere to the exercise behavior and maintain the stability of that behavior.

Another important finding is that controlled motivation negatively affected behavioral intention while it positively affected usage behavior in the context of compelling college students to use sports apps. However, previous studies have shown that controlled motivation has no significant effect on both exercise intention and behavior [44, 45]. The reasons may be that the mandatory behavior of the school restricts students' freedom to choose extracurricular physical exercises to a certain extent. According to reactance theory, the restriction on freedom of behavior is fundamentally a threat [58, 59], which results in students' disgust and dissatisfaction with the use of sports apps, leading to a negative effect on behavioral intention. Contrastingly, to promote students' running exercise, the schools have set the goal of using sports apps for students (specifying the number of runs and total mileage using sports apps during the semester). A study on the progress of goals [60] showed that controlled motivation promotes the achievement of goals in the short term, especially in contexts that often provide important clues for achieving specific goals and has a greater impact on goals progress. Physical education teachers' supervision and persuasion in class and the running behavior of surrounding classmates using the sports apps provide important clues for the achievement of students' running goals. Therefore, controlled motivation positively affects the usage behavior of sports apps in the mandatory situation of this study. However, the influence of controlled motivation on the behavior of using sports apps may disappear when students' running goals are achieved. Therefore, schools need to develop strategies to facilitate the internalization of controlled motivation into autonomous motivation; that is, to facilitate the transformation of “mandatory exercise” into “active exercise” by students. Legate et al. [59] showed that autonomy support information and enhanced understanding of mandatory behavior goals would increase autonomous motivation and decrease controlled motivation. Therefore, the relevant departments of the school should make students understand the original purpose of the school's mandatory behavior through persuasive education and other means, make them aware of the benefits and necessity of exercise, and enhance their initiative and sense of identity. Concurrently, physical education teachers should actively encourage and guide students, but prohibit the transmission of threats, coercion, and other negative information, and try their best to reduce or avoid triggering students' resistance tendency. The above strategies can gradually improve students' autonomous motivation level, promote the internalization of controlled motivation, and strive to make students' exercise behavior last longer.

Furthermore, facilitating conditions had no significant effect on the usage behavior of the sports apps in mandatory situations. Facilitating conditions are defined as the degree that an individual believes that an organizational and technical infrastructure exists to support use of the system [26]. The current technical infrastructure that supports sports apps is very well developed. College students are familiar with the operation of smartphones and apps and can use them proficiently without training or guidance. Additionally, Venkatesh et al. [26] believed that facilitating conditions have a significant effect on usage behavior only when it is moderated by age and experience. These two moderator variables were not included in this study because the age gap and operational experience were insufficient to make any difference in the results. Therefore, the effect of facilitating conditions on usage behavior is not significant.

Concerning moderator variable, although gender had a moderating effect in UTAUT, this gender difference will gradually disappear with the development of the economy and information technology [26]. Owing to the widespread use of smart phones and college students' proficiency with app operation, the results indicate that there are no significant gender differences in the effects of performance expectancy, effort expectancy, and social influence on the intention to use sports apps.

### 4.2. Strengths, Limitations, and Future Research

To the best of our knowledge, this study is the first to explore the influencing factors of college students' acceptance and use of sports apps in mandatory situations from the perspectives of technical acceptance and motivation. The results profoundly contribute to the sports apps adoption literature and support technical developers and schools in formulating appropriate improvement strategies and policies. These are helpful to fully exploit the beneficial role of new media technology in intervening with college students' physical exercise habits and physical health improvement.

The study has several limitations. First, this study is cross-sectional and thus cannot demonstrate changes in intention and behavior over time. Second, the survey was conducted only in China; hence, the findings may not be applicable to other countries with different cultures and levels of acceptance of sports apps. Third, this study employed a non-probability sampling method, and participants were limited to Liaoning University of Technology; therefore, the generalizability of the findings may have some limitations.

In future research, the following should be considered. First, longitudinal studies should be considered to provide a more comprehensive understanding of the short-, medium-, and long-term effects of mandating college students to use sports apps. Second, to provide more evidence, future relevant studies should be conducted in different cultural backgrounds. Third, future research can further strengthen the study of the influence of psychological factors such as attitude, satisfaction, and emotion to gain a more comprehensive understanding of the factors influencing college students' use of sports apps in mandatory situations.

## 5. Conclusions

Sports apps are an important technical tool to help college students develop exercise habits and improve their physical health. This study constructs a research model based on UTAUT and SDT to explore the factors influencing college students' use of sports apps in mandatory situations, using the “campus running” app as a case study. The research model can explain 66% of the variance in behavioral intention and 30% of the variance in usage behavior. Concerning the influencing factors of students' intention to use sports apps, performance expectancy, effort expectancy, social influence, and autonomous motivation are important positive factors of behavioral intention, while controlled motivation is a negative factor. Concerning the influencing factors of usage behavior, behavioral intention, autonomous motivation, and controlled motivation are positive factors of usage behavior, among which autonomous motivation is the most important influencing factor. However, the influence of facilitating conditions on usage behavior is not significant. The results profoundly contribute to the sports apps adoption literature, and help technical developers and schools to formulate corresponding improvement strategies and policies to further promote the role sports apps play in college students' exercise behavior.

## Figures and Tables

**Figure 1:** Unified theory of acceptance and use of technology (Source: Venkatesh et al., [26]).

**Figure 2:** Research model of sports apps usage behavior in mandatory situations. Note: The dotted line indicates that the research hypothesis is not significant.

**Figure 3:** Model results. Note: ∗*p <0.05,*∗∗*p <0.01,*∗∗∗*p <0.001.* The dotted line indicates that the influence is not significant.

**Table 1:** Descriptive statistics of participants' characteristics. (*N* =249).

Characteristics	Frequency (n)	Percent (%)
Age (mean ± SD)	19.28 ± 1.02	
*Gender*		
Male	104	41.77
Female	145	58.23
*Degree*		
Freshman	132	53.01
Sophomore	117	46.99
*Usage behavior*		
1-3 times/week	75	30.12
4-5 times/week	120	48.19
6-7 times/week	54	21.69

**Table 2:** Descriptive statistics of the questionnaire.

Constructs and items	Skewness	Kurtosis	Factors loading
Performance expectancy			
PE1. Using “campus running” app could inspire you to keep doing physical activity.	-0.76	-0.34	0.78
PE2. Using “campus running” app could contribute to maintaining physical fitness.	-0.26	-0.53	0.82
PE3. Using “campus running” app could contribute to maintaining good mental health.	-0.13	-0.55	0.85
Effort expectancy			
EE1. You can quickly master how to use “campus running” app.	0.08	-0.85	0.83
EE2. You can be proficient with using “campus running” app.	0.23	-0.49	0.80
EE3. Using “campus running” app is not difficult for you.	-0.02	-0.61	0.80
Social influence			
SI1. People who are important to me think that I should use the “campus running” app.	0.17	-0.63	0.78
SI2. People who influence my behavior think that I should use the “campus running” app.	0.02	-0.70	0.84
SI3. People whose opinions that I value prefer that I use the “campus running” app.	0.42	-0.84	0.79
Facilitating conditions			
FC1. I have the resources necessary to use the “campus running” app.	-0.23	1.17	0.86
FC2. I have the knowledge necessary to use the “campus running” app.	-0.19	0.00	0.78
FC3. The “campus running” app is compatible with other technologies I use.	0.09	0.54	0.93
Autonomous motivation			
AM1. I value the benefits of using the “campus running” app.	-0.06	-0.75	0.80
AM2. It's important to me to use the “campus running” app regularly.	0.00	-0.94	0.76
AM3. I use the “campus running” app because it is consistent with life goals.	0.49	0.38	0.80
AM4. I consider using the “campus running” app consistent with my values.	0.16	-0.02	0.79
AM5. I use the “campus running” app because it's fun.	0.29	0.02	0.75
AM6. I get pleasure/satisfaction from using the “campus running” app.	-0.31	-0.95	0.54
Controlled motivation			
CM1. I use the “campus run” app because other people say I should.	-0.03	-0.70	0.82
CM2. I use the “campus run” app because I feel under pressure from others.	0.13	-0.58	0.80
CM3. I feel guilty when I do not use the “campus run” app.	0.07	-0.62	0.74
CM4. I feel ashamed when I miss using the “campus running” app.	0.00	-0.55	0.67
Behavioral intention			
BI1. How many times do you intend to use the “campus running” app in the next week?	-0.32	-0.30	0.79
BI2. How many times do you plan to use the “campus running” app in the next week?	-0.13	-0.65	0.83
BI3. How many times do you try to use the “campus running” app in the next week?	-0.11	-0.73	0.86
Usage behavior			
These usage data were exported directly from the app's data monitoring background.	0.18	-0.72	1.00

**Table 3:** Construct reliability, convergent and Fornell-Larcker criterion.

Constructs	*α*	CR	AVE	PE	EE	SI	FC	AM	CM	BI
PE	0.74	0.85	0.66	**0.81**						
EE	0.74	0.85	0.65	0.47	**0.81**					
SI	0.72	0.84	0.64	0.52	0.64	**0.80**				
FC	0.83	0.89	0.74	0.32	0.31	0.34	**0.86**			
AM	0.79	0.88	0.70	0.48	0.78	0.70	0.43	**0.84**		
CM	0.77	0.90	0.81	0.49	0.62	0.69	0.34	0.69	**0.90**	
BI	0.77	0.87	0.68	0.64	0.71	0.66	0.36	0.69	0.55	**0.83**

Note: *α* = Cronbach's alpha; CR = composite reliability; AVE = average variance extracted; PE = performance expectancy; EE = effort expectancy; SI = social influence; FC = facilitating conditions; AM = autonomous motivation; CM = controlled motivation; BI = behavioral intention; numbers in bold = square root of AVE.

**Table 4:** The cross loadings.

Items	PE	EE	SI	FC	AM	CM	BI
PE_1	**0.78**	0.26	0.26	0.22	0.30	0.23	0.48
PE_2	**0.82**	0.38	0.51	0.33	0.43	0.49	0.53
PE_3	**0.85**	0.48	0.49	0.22	0.45	0.47	0.54
EE_1	0.38	**0.83**	0.47	0.26	0.62	0.51	0.55
EE_2	0.30	**0.80**	0.55	0.24	0.64	0.52	0.51
EE_3	0.43	**0.80**	0.53	0.25	0.63	0.48	0.64
SI_1	0.49	0.54	**0.78**	0.27	0.58	0.77	0.56
SI_2	0.40	0.52	**0.84**	0.26	0.57	0.48	0.55
SI_3	0.36	0.48	**0.79**	0.28	0.52	0.40	0.48
FC_1	0.28	0.26	0.26	**0.86**	0.37	0.29	0.32
FC_2	0.27	0.21	0.26	**0.78**	0.29	0.28	0.24
FC_3	0.28	0.32	0.34	**0.93**	0.42	0.32	0.35
AM_1	0.44	0.68	0.58	0.35	**0.85**	0.56	0.71
AM_2	0.40	0.69	0.64	0.36	**0.87**	0.62	0.54
AM_3	0.36	0.57	0.54	0.39	**0.79**	0.55	0.42
CM_1	0.47	0.62	0.62	0.32	0.68	**0.92**	0.52
CM_2	0.42	0.48	0.63	0.30	0.54	**0.88**	0.46
BI_1	0.54	0.47	0.50	0.32	0.42	0.40	**0.79**
BI_2	0.52	0.58	0.53	0.27	0.56	0.46	**0.83**
BI_3	0.53	0.67	0.61	0.31	0.69	0.48	**0.86**

Note: Numbers in bold = indicator's outer loadings on the associated construct.

**Table 5:** Path coefficients and hypotheses testing.

Hypotheses	Relationship	Std. beta	*t*-value	*p*-value	*f* ^2^	Decision
H1	PE → BI	0.33	6.55	0.000	0.21	Supported
H2	EE → BI	0.33	5.20	0.000	0.12	Supported
H3	SI → BI	0.22	3.76	0.000	0.06	Supported
H4	FC → UB	-0.03	0.39	0.694	0.00	Not supported
H5	BI → UB	0.21	2.75	0.006	0.03	Supported
H7a	AM → BI	0.19	2.64	0.008	0.03	Supported
H7b	AM →UB	0.27	2.76	0.006	0.04	Supported
H8a	CM → BI	-0.10	1.96	0.050	0.01	Not supported
H8b	CM → UB	0.16	2.12	0.034	0.02	Not supported

Note: UB = usage behavior.

## Data Availability

The data used to support the findings of this study are available from the corresponding author upon request.
